The article "Identification and analysis of genes associated with papillary thyroid carcinoma by bioinformatics methods" was published in 2019. Journal: Biosci Rep.

# Identification and analysis of genes associated with papillary thyroid carcinoma by bioinformatics methods

**DOI:** 10.1042/BSR20190083

**Published:** 2019-04-02

**Authors:** Shulong Zhang, Quan Wang, Qi Han, Huazhong Han, Pinxiang Lu

**Affiliations:** Department of General Surgery, Xuhui District Central Hospital of Shanghai, Shanghai 200031, China

**Keywords:** Key gene, Papillary thyroid carcinom, Signaling pathway, Survival analysis

## Abstract

The molecular mechanism of the occurrence and development of papillary thyroid carcinoma (PTC) has been widely explored, but has not been completely elucidated. The present study aimed to identify and analyze genes associated with PTC by bioinformatics methods. Two independent datasets were downloaded from Gene Expression Omnibus (GEO) database. The differentially expressed genes (DEGs) between PTC tissues and matched non-cancerous tissues were identified using GEO2R tool. The common DEGs in the two datasets were screened out by VennDiagram package, and analyzed by the following tools: KOBAS, Database for Annotation, Visualization, and Integrated Discovery (DAVID), Search tool for the retrieval of interacting genes/proteins (STRING), UALCAN and Gene expression profiling interactive analysis (GEPIA). A total of 513 common DEGs, including 259 common up-regulated and 254 common down-regulated genes in PTC, were screened out. These common up-regulated and down-regulated DEGs were most significantly enriched in cytokine–cytokine receptor interaction and metabolic pathways, respectively. Protein–protein interactions (PPI) network analysis showed that the up-regulated genes: *FN1, SDC4, NMU, LPAR5* and the down-regulated genes: *BCL2* and *CXCL12* were key genes. Survival analysis indicated that the high expression of *FN1* and *NMU* genes significantly decreased disease-free survival of patients with thyroid carcinoma. In conclusion, the genes and pathways identified in the current study will not only contribute to elucidating the pathogenesis of PTC, but also provide prognostic markers and therapeutic targets for PTC.

## Introduction

Papillary thyroid carcinoma (PTC) is the most common subtype of thyroid malignancy, and accounts for approximately 75% of all thyroid cancers [1]. Although PTC has been reported as a curable malignancy with more than 90% 10-year survival, the incidence of PTC had been increasing and a subset of patients died of the disease due to local recurrence or distant metastasis [2–4]. Therefore, the molecules involved in the occurrence and development of PTC needs to be explored, which will contribute to the finding of prognostic markers and therapeutic targets of PTC.

Previous studies have made an important contribution to revealing the pathogenesis of PTC [5–7]. For instance, Dong et al. [5] found that estrogen could induce the metastatic potential of PTC cells through estrogen receptor α and β. Yin et al. [6] found that *miR-195* was down-regulated in PTC. Overexpression of *miR-195* could significantly inhibit the growth and metastasis of PTC cells by targeting CCND1 and FGF2. Shen et al. [7] found that lncRNA PROX1-AS1 could promote the proliferation, invasion and migration of PTC cells and might act as a potential target for PTC therapy. However, the above findings were obtained based on molecular biological methods, such as Western blot, immunohistochemistry and dual-luciferase reporter assay system. These methods were often used to explore the specific function of a certain molecule in disease, and could not observe the overall change of molecules in cells. With the development of high-throughput molecular detection technology, an increasing number of gene expression profiling data can be generated by microarray or RNA-seq. By bioinformatic analysis of these data, researchers found many novel genes associated with disease initiation and progression [8–10]. In the current study, we utilized various bioinformatics methods to mine high-throughput gene expression data of PTC and normal thyroid tissues, and identified several key genes associated with PTC, such as *FN1, SDC4, NMU, LPAR5, BCL2* and *CXCL12*, which might act as prognostic markers and therapeutic targets for PTC.

## Materials and methods

### Microarray data

High-throughput gene expression data of PTC and normal thyroid tissues from two independent datasets (GSE3467 and GSE29265) were obtained from Gene Expression Omnibus (GEO, https://www.ncbi.nlm.nih.gov/geo/). Thereinto gene expression profiling data of nine paired PTC and normal thyroid tissues were from GSE3467, which were generated by the GPL570 platform (Affymetrix Human Genome U133 Plus 2.0 Array) and contributed by He et al. [11]. Other data including 20 paired PTC and noncancerous tissues were from GSE29265, which were generated by the GPL570 platform (Affymetrix Human Genome U133 Plus 2.0 Array) and contributed by Tomas et al. (https:www.ncbi.nlm.nih.gov/geo/query/acc.cgi?acc=GSE29265).

### Identification of differentially expressed genes

GEO2R tool (https://www.ncbi.nlm.nih.gov/geo/geo2r/) was used to identify differentially expressed genes (DEGs) in PTC tissues compared with matched non-cancerous tissues. The *t*-test and Benjamini–Hochberg method were used to calculate the *P*-value and FDR, respectively. The DEGs were screened out according to adjusted *P*-value <0.05 and |logFC| ≥1. The common DEGs in the two datasets were screened out by VennDiagram package [12].

### Kyoto encyclopedia of genes and genomes pathway enrichment analysis

KOBAS 3.0 (http://kobas.cbi.pku.edu.cn/) is an online tool for gene/protein functional annotation and gene set functional enrichment [13]. For enrichment analysis, KOBAS 3.0 can accept either gene list or gene expression data as input, and generates enriched gene sets, corresponding name, *P*-value or a probability of enrichment and enrichment score based on results of multiple methods. To identify key pathways implicating PTC, we conducted Kyoto Encyclopedia of Genes and Genomes (KEGG) pathway enrichment of common DEGs by using KOBAS 3.0. A corrected *P*-value <0.05 was considered significant.

### Protein–protein interactions network and module analysis

The Search Tool for the Retrieval of Interacting Genes/Proteins (STRING) database (http://string-db.org/) consolidates known and predicted protein–protein association data for a large number of organisms, which contributes to uncovering the direct (physical) and indirect (functional) relationships of DEGs [14]. In the present study, Protein–protein interactions (PPI) network of common DEGs were constructed by the latest STRING v10.5 database based on a minimum required interaction score 0.7. PPI network with the most number of nodes were visualized by Cytoscape v3.3.0 software. Key nodes (genes) in the PPI network were screened out according to node degree >10. Furthermore, a Cytoscape App, Molecular Complex Detection (MCODE v1.4.1) with K-Core >4 was used to detect densely connected regions (modules) in the PPI network that might represent molecular complexes [15]. Database for Annotation, Visualization, and Integrated Discovery (DAVID) v.6.8 (https://david.ncifcrf.gov/tools.jsp) can annotate input genes, classify gene functions, identify gene conversions and carry out gene ontology (GO) term analysis. Thus, the DAVID was used to annotate genes in each densely connected region and perform GO term enrichment, which helped reveal the biological function of each densely connected region [16,17]. FDR value <0.05 was considered significant.

### Validation of the expression level of key genes in PPI network

UALCAN (http://ualcan.path.uab.edu/) is a user-friendly, interactive web resource for analyzing transcriptome data of cancers from The Cancer Genome Atlas (TCGA) [18]. In the current study, the online tool was used to validate the expression level of key genes in PPI network.

### Association of key genes expression with survival of patients with thyroid carcinoma

Gene Expression Profiling Interactive Analysis tool (GEPIA, http://gepia.cancer-pku.cn/) could deliver fast and customizable functionalities based on TCGA and GTEx data [19], including differential expression analysis, profiling plotting, correlation analysis, patient survival analysis, similar gene detection and dimensionality reduction analysis. In the current study, GEPIA was utilized to explore the association of key gene expression with disease-free survival (DFS) of patients with thyroid carcinoma. Patients were grouped into high expression group and low expression group according to the median value of gene expression. *P*(HR)-value <0.05 was considered statistically significant.

### Analysis of the main functional regions of proteins encoded by key genes

UniProt provided a comprehensive and high-quality resource of protein sequences and their annotations, such as functional region, subcellular location, structure and so on, and can be freely accessed via the website at http://www.uniprot.org/ [20]. In the current study, UniProt was utilized to summarize the main functional regions of proteins encoded by key genes.

## Results

### Identification of DEGs

For GSE3467 dataset, a total of 771 DEGs, including 373 up-regulated and 398 down-regulated genes in PTC, were identified. For GSE29265 dataset, a total of 847 DEGs, including 417 up-regulated genes and 430 down-regulated genes in PTC, were screened out. Intersection analysis of the two datasets showed 513 common DEGs, including 259 common up-regulated and 254 common down-regulated genes in PTC (Figure 1 and Supplement). KEGG pathway enrichment analysis indicated that these common up-regulated genes were significantly enriched in 43 pathways. The top ten pathways included ‘Cytokine–cytokine receptor interaction’, ‘Pathways in cancer’, ‘p53 signaling pathway’, ‘Small cell lung cancer’, ‘Proteoglycans in cancer’, ‘Transcriptional misregulation in cancer’, ‘Focal adhesion’, ‘ECM–receptor interaction’, ‘Cell adhesion molecules’ and ‘Complement and coagulation cascades’ (Figure 2A). These common down-regulated genes were significantly enriched in 27 pathways. The top ten pathways included ‘Metabolic pathways’, ‘Insulin resistance’, ‘Adipocytokine signaling pathway’, ‘Tyrosine metabolism’, ‘AMPK signaling pathway’, ‘Hedgehog signaling pathway’, ‘Retinol metabolism’, ‘Thyroid hormone synthesis’, ‘Fructose and mannose metabolism’ and ‘Cytokine–cytokine receptor interaction’ (Figure 2B).

**Figure 1:** The common differentially expressed genes in the two datasets (**A**) Common up-regulated genes; (**B**) common down-regulated genes.

**Figure 2:** The top ten KEGG pathways enriched by common differentially expressed genes (**A**) common up-regulated genes; (**B**) common down-regulated genes.

### PPI network of common DEGs

The PPI network of common DEGs, including 170 nodes (genes) and 328 edges (interactions), were constructed (Figure 3A). The degree centrality analysis showed that *FN1, BCL2, CXCL12, SDC4, NMU* and *LPAR5* genes were key genes. Therein the expression levels of *FN1, SDC4, NMU* and *LPAR5* genes were up-regulated in PTC. The expression levels of *BCL2* and *CXCL12* genes were down-regulated in PTC (Figure 3B). In addition, two significant modules were identified in PPI network (Figure 4A,B). Due to the limited number of genes in each module, we furtherly analyzed each module as a whole. Genes in Module 1 were significantly enriched in ‘G-protein coupled receptor signaling pathway’, ‘Cell chemotaxis’, ‘Negative regulation of leukocyte tethering or rolling’, ‘Chemokine activity’. Genes in Module 2 were significantly enriched in ‘Extracellular region’, ‘Endoplasmic reticulum lumen’, ‘Collagen trimer’, ‘Platelet degranulation’, ‘Platelet alpha granule lumen’, ‘Collagen catabolic process’, ‘Extracellular matrix organization’, ‘Proteinaceous extracellular matrix’, ‘Extracellular matrix’ and ‘Protease binding’ (Figure 4C).

**Figure 3:** Construction and analysis of PPI network of common differentially expressed genes PPI network plot (**A**): red and light blue nodes indicate up- and down- regulated genes, respectively; the node size indicates the node degree. Key nodes in PPI network (**B**): a node degree is defined as the number of other nodes connected to the node.

**Figure 4:** Identification and analysis of significant modules in PPI network Two significant modules in PPI network (**A**): module 1 network; (**B**): module 2 network; (**C**): gene ontology enrichment results of different modules. The cut-off value of ‘significant’ modules is K-Core >4).

### Validation of the expression level of key genes in PPI network

TCGA data analysis showed that *FN1, SDC4, NMU* and *LPAR5* genes were significantly up-regulated in PTC, and *BCL2* and *CXCL12* genes were significantly down-regulated in PTC, which were consistent with the results of microarray analysis (Figure 5).

**Figure 5:** The expression level of key genes in papillary thyroid carcinoma from TCGA

### Association of key genes expression with survival of patients with thyroid carcinoma

Survival analysis based on TCGA data showed that the expression levels of *SDC4, BCL2, CXCL12* and *LPAR5* genes were not associated with DFS of patients with thyroid carcinoma; however, the high expression of *FN1* and *NMU* genes significantly decreased DFS of patients with thyroid carcinoma (Figure 6).

**Figure 6:** The association of the expression level of key genes with DFS of patients with thyroid carcinoma The association of the expression level of key genes with DFS of patients with thyroid carcinoma based on TCGA [*P*(HR) value <0.05 was considered to be associated with DFS].

### Analysis of the main functional regions of proteins encoded by key genes

Information of the main functional regions of proteins encoded by *FN1* and *CXCL12* genes was obtained from UniProt and summarized in Table 1. The protein encoded by *FN1* gene contained eight main functional regions, including 52–272 aa (fibrin- and heparin-binding 1), 308–608 aa (collagen-binding), 464–477 aa (critical for collagen binding), 1267–1540 aa (cell-attachment), 1721–1991 aa (heparin-binding 2), 1813–1991 aa (binds to FBLN1), 1992–2102 aa [connecting strand 3 (CS-3) (V region)] and 2206–2337 aa (fibrin-binding 2). The protein encoded by *CXCL12* gene had five main functional regions, including 29–33 aa (receptor and heparin binding), 39–41 aa (receptor binding), 41–51 aa (heparin binding), 48–50 aa (receptor binding) and 60–70 aa (receptor binding).

**Table 1:** Summary of the main functional regions of proteins encoded by key genes

Gene name	Protein name	Uniport entry	Organism	Length	Main functional regions	
					Regions	Description
FN1	Fibronectin	P02751	Homo sapiens	2386	52–272	Fibrin- and heparin-binding 1
					308–608	Collagen-binding
					464–477	Critical for collagen binding
					1267–1540	Cell-attachment
					1721–1991	Heparin-binding 2
					1813–1991	Binds to FBLN1
					1992–2102	Connecting strand 3 (CS-3) (V region)
					2206–2337	Fibrin-binding 2
SDC4	Syndecan-4	P31431	Homo sapiens	198	-	-
NMU	Neuromedin-U	P48645	Homo sapiens	174	-	-
LPAR5	Lysophosphatidic acid receptor 5	Q9H1C0	Homo sapiens	372	-	-
BCL2	Apoptosis regulator Bcl-2	P10415	Homo sapiens	239	-	-
CXCL12	Stromal cell-derived factor 1	P48061	Homo sapiens	93	29–33	Receptor and heparin binding
					39–41	Receptor binding
					41–51	Heparin binding
					48–50	Receptor binding
					60–70	Receptor binding

## Discussion

In the present study, we analyzed gene expression profiling data of 29 paired PTC tissues and corresponding non-cancerous tissues from two independent datasets, and found 513 common DEGs, including 259 common up-regulated and 254 common down-regulated genes in PTC. Pathway enrichment analysis indicated that these common up-regulated and down-regulated DEGs were most significantly enriched in cytokine–cytokine receptor interaction and metabolic pathways, respectively. PPI network analysis showed that *FN1, SDC4, NMU, LPAR5, BCL2* and *CXCL12* genes had high degree centrality, suggesting that these genes might play an important role in the occurrence or development of PTC. In order to validate the expression level of these key genes, we further analyzed related data in TCGA. Results indicated that *FN1, SDC4, NMU* and *LPAR5* genes were significantly up-regulated in PTC, and *BCL2* and *CXCL12* genes were significantly down-regulated in PTC, which were consistent with the results of microarray analysis. In addition, survival analysis showed that the high expression of *FN1* and *NMU* genes significantly decreased DFS of patients with thyroid carcinoma.

By reviewing the previous studies, we found that these crucial genes were involved in the initiation and progress of various cancers [21–28]. For instance, Sponziello et al. [21] found that FN1 expression was significantly overexpressed in PTC tissues compared with normal tissues. Silencing of FN1 significantly reduced proliferation, adhesion, migration and invasion of PTC cells. Chen et al. [22] observed that *SDC4* gene silencing not only favored human PTC cell apoptosis, but also inhibited epithelial mesenchymal transition via Wnt/β-catenin pathway. Zhu et al. [23] confirmed that CXCL12 could stimulate the invasion and migration of K1 cells overexpressing CXCR4, but did not affect K1 cells overexpressing CXCR7, which suggested that CXCL12 function in cancer depended on the assistance of other molecules. In addition, results of Zhang’s study suggested that *CXCL12* down-regulation in PTC might be caused by promoter hypermethylation [24]. Although the specific biological functions of *BCL2* and *LPAR5* genes in PTC had not been explored directly by molecular biology methods, data mining based on bioinformatics tools had also confirmed that *BCL2* gene was down-regulated in PTC [25], and *LPAR5* gene was up-regulated in thyroid cancer [26]. To the best of our knowledge, *NMU* gene had not been identified as key genes in PTC so far. However, the promotion effect of *NMU* gene on other cancers had been reported [27,28]. For instance, Lin et al. [27] found that NMU signaling promoted endometrial cancer cell progression by modulating adhesion signaling. Martinez et al. [28] found that overexpression of NMU resulted in up-regulation of epithelial–mesenchymal transition markers and expanded the cancer stem cell phenotype in HER2-positive breast cancer. Furthermore, the current result showed that the high expression of *NMU* gene significantly decreased DFS of patients with thyroid carcinoma. Thus, the specific functions of *NMU* in PTC were worth to be further explored.

In conclusion, our study identified several key genes (*FN1, SDC4, NMU, LPAR5, BCL2* and *CXCL12*) and signaling pathways (cytokine–cytokine receptor interaction and metabolic pathways) associated with PTC, which might act as prognostic markers and therapeutic targets for PTC. However, further experimental studies are still required to confirm the functions of identified genes, such as *BCL2, LPAR5* and *NMU*.

## Supporting information

**Supplemental Table S1:** 

## Abbreviations

BCL2: BCL2 apoptosis regulator
CCND1: Cyclin D1
CXCL12: C-X-C motif chemokine ligand 12
DAVID: Database for annotation, visualization, and integrated discovery
DEG: differentially expressed gene
DFS: disease-free survival
ECM: Extracellular matrix
FDR: False discovery rate
FGF2: Fibroblast growth factor 2
FN1: Fibronectin 1
GEO: Gene expression omnibus
GEPIA: Gene expression profiling interactive analysis
GO: gene ontology
GTEx: Genotype-Tissue Expression
HR: Hazard ratio
KEGG: Kyoto encyclopedia of genes and genomes
LPAR5: Lysophosphatidic acid receptor 5
NMU: Neuromedin U
PPI: Protein–protein interaction
PTC: papillary thyroid carcinoma
SDC4: Syndecan 4
STRING: Search tool for the retrieval of interacting genes/proteins
TCGA: The Cancer Genome Atlas
